The article "Nanosized TiO2-Induced Reproductive System Dysfunction and Its Mechanism in Female Mice" was retracted in 2024. Reasons: errors in the analysis; duplicated text; overlap with earlier publications; unreliable results or conclusions.

# Nanosized TiO_2_-Induced Reproductive System Dysfunction and Its Mechanism in Female Mice

**DOI:** 10.1371/journal.pone.0059378

**Published:** 2013-04-02

**Authors:** Xiaoyang Zhao, Yuguan Ze, Guodong Gao, Xuezi Sang, Bing Li, Suxin Gui, Lei Sheng, Qingqing Sun, Jie Cheng, Zhe Cheng, Renping Hu, Ling Wang, Fashui Hong

**Affiliations:** Medical College, Soochow University, Suzhou, People’s Republic of China; "Mario Negri" Institute for Pharmacological Research, Italy

## Abstract

Recent studies have demonstrated nanosized titanium dioxide (nano-TiO_2_)-induced fertility reduction and ovary injury in animals. To better understand how nano-TiO_2_ act in mice, female mice were exposed to 2.5, 5, and 10 mg/kg nano-TiO_2_ by intragastric administration for 90 consecutive days; the ovary injuries, fertility, hormone levels, and inflammation-related or follicular atresia-related cytokine expression were investigated. The results showed that nano-TiO_2_ was deposited in the ovary, resulting in significant reduction of body weight, relative weight of ovary and fertility, alterations of hematological and serum parameters and sex hormone levels, atretic follicle increases, inflammation, and necrosis. Furthermore, nano-TiO_2_ exposure resulted in marked increases of insulin-like growth factor-binding protein 2, epidermal growth factor, tumor necrosis factor-α, tissue plasminogen activator, interleukin-1β, interleukin -6, Fas, and FasL expression, and significant decreases of insulin-like growth factor-1, luteinizing hormone receptor, inhibin α, and growth differentiation factor 9 expression in mouse ovary. These findings implied that fertility reduction and ovary injury of mice following exposure to nano-TiO_2_ may be associated with alteration of inflammation-related or follicular atresia-related cytokine expressions, and humans should take great caution when handling nano-TiO_2_.

## Introduction

The manufacture and application of various synthetic nanoparticles are expanding at a rapid rate, and therefore increased environmental and occupational exposures of these materials seem inevitable. Nanosized titanium dioxide (nano-TiO_2_) presents various uses in industry, in commerce such as cosmetics, sunscreen, toothpaste, food additives and paints, and even in the treatment of contaminated environments [1]–[4]. However, toxicological studies suggested that nano-TiO_2_ had adverse effects on human health and environmental species. The bio-safety of nano-TiO_2_ is still an argumentative issue.

Toxicological properties of nano-TiO_2_ have been studied in kidney [5]–[8], and brain [9]–[14] of animals. Especially, recent studies demonstrated that exposure to nano-TiO_2_ resulted in toxicity in reproductive system. For example, nano-TiO_2_ can reduce sperm density and motility, increase sperm abnormality and germ cell apoptosis of male mice *in vivo* [15], inhibit follicle development and oocyte maturation of rat *in vitro* [16], affect development, reproduction, and locomotion behavior of Caenorhabditis elegans [17], induce genotoxicity and cytotoxicity in Chinese hamster ovary cells *in vitro* [18], and impair zebrafish reproduction [19]. Nano-TiO_2_ was also administered subcutaneously to pregnant mice and transferred to the offspring and impaired the genital and cranial nerve systems of the male mice offspring [20]. However, the mechanisms of nano-TiO_2_–induced toxicity in reproductive system have yet to be understood. The present study was designed to investigate histopathological changes of ovary, fertility, and sex hormone levels in female mice following exposure to 2.5, 5, and 10 mg/kg body weight TiO_2_ NPs 90 consecutive days. Furthermore, the inflammation-related or follicular atresia-related cytokine expressions were also examined by real time RT-PCR and ELISA after female mice exposure to nano-TiO_2_. Our results showed that nano-TiO_2_ can induce ovarian dysfunction measured by histological assessment, mating rate, pregnancy rate, number of newborns, and sex hormone levels. Nano-TiO_2_ also significantly altered the inflammation-related or follicular atresia-related cytokine expressions in the mouse ovary.

## Materials and Methods

### Preparation and Characterization of Nano-TiO_2_

Nanoparticulate anatase TiO_2_ of the synthesis and characterization of nano-TiO_2_ was described in our previous reports [13], [21]. In a typical experiment, 1 mL of Ti (OC4H9)4 was dissolved in 20 ml of anhydrous isopropanol, and was added dropwise to 50 mL of double-distilled water that was adjusted to pH 1.5 with nitric acid under vigorous stirring at room temperature. The temperature of the solution was then raised to 60°C, and maintained for 6 hours to promote better crystallization of nanoparticulate TiO_2_ particles. Using a rotary evaporator, the resulting translucent colloidal suspension was evaporated yielding a nanocrystalline powder. The obtained powder was washed three times with isopropanol, and then dried at 50°C until the evaporation of the solvent was complete. A 0.5% w/v hydroxypropylmethylcellulose (HPMC) K4M was used as a suspending agent. TiO_2_ powder was dispersed onto the surface of 0.5% w/v HPMC solution, and then the suspending solutions containing TiO_2_ particles were treated ultrasonically for 15–20 min and mechanically vibrated for 2 min or 3 min.

The particle sizes of both the powder and nanoparticle suspended in 0.5% w/v HPMC solution after incubation for 24 h (5 mg/mL) were determined using a TecnaiG220 transmission electron microscope (TEM) (FEI Co., USA) operating at 100 kV, respectively. In brief, particles were deposited in suspension onto carbon film TEM grids, and allowed to dry in air. Mean particle size was determined by measuring more than 100 individual particles that were randomly sampled. X-ray-diffraction (XRD) patterns were obtained at room temperature with a MERCURY CCD diffractometer (MERCURY CCD Co., Japan) using Ni-filtered Cu Kα radiation. The surface area of each sample was determined by Brunauer–Emmett–Teller (BET) adsorption measurements on a Micromeritics ASAP 2020M+ C instrument (Micromeritics Co., USA). The average aggregate or agglomerate size of the TiO_2_ NPs after incubation in 0.5% w/v HPMC solution for 24 h (5 mg/mL) was measured by dynamic light scattering (DLS) using a Zeta PALS+BI-90 Plus (Brookhaven Instruments Corp., USA) at a wavelength of 659 nm. The scattering angle was fixed at 90°. The average particle sizes of powdered nano-TiO_2_ that suspended in 0.5% w/v hydroxypropylmethylcellulose (HPMC) K4M solvent after 24 h incubation ranged from 5 to 6 nm. The surface area of the sample was 174.8 m^2^/g. The mean hydrodynamic diameter of TiO_2_ NP in HPMC solvent ranged from 208 to 330 nm (mainly 294 nm), and the zeta potential after 24 h incubation was 9.28 mV, respectively [13].

### Ethics Statement

All experiments were conducted during the light phase, and were approved by the Animal Experimental Committee of the Soochow University(Grant 2111270) and in accordance with the National Institutes of Health Guidelines for the Care and Use of Laboratory Animals(NIH Guidelines).

### Animals and Treatment

CD-1 (ICR) female mice were used in this study. 400 CD-1 (ICR) female mice and 40 CD-1 (ICR) male mice (18±2 g) were purchased from the Animal Center of Soochow University (China). All mice were housed in stainless steel cages in a ventilated animal room. Room temperature of the housing facility was maintained at 24±2°C with a relative humidity of 60±10% and a 12-h light/dark cycle in Animal Center of Soochow University (China). Distilled water and sterilized food were available for mice *ad libitum*. Prior to dosing, the mice were acclimated to this environment for 5 days.

A 0.5% HPMC was used as a suspending agent. Nano-TiO_2_ powder was dispersed onto the surface of 0.5%, w/v HPMC, and then the suspending solutions containing TiO_2_ NPs were treated by ultrasonic for 30 min and mechanically vibrated for 5 min. About the dose selection in this study, we consulted the report of World Health Organization in 1969. According to the report, LD50 of TiO_2_ for rats is larger than 12,000 mg/kg body weight (BW) after oral administration. In addition, the quantity of TiO_2_ nanoparticles does not exceed 1% by weight of the food according to the Federal Regulations of US Government. In the present study, we selected 2.5, 5, and 10 mg/kg BW TiO_2_ NPs exposed to mice by intragastric administration every day. They were equal to about 0.15–0.7 g TiO_2_ NPs of 60–70 kg body weight for humans with such exposure, which were relatively safe doses. For the experiment, the female mice were randomly divided into four groups (each group N = 100), including a control group (treated with 0.5% w/v HPMC) and three experimental groups (2.5, 5, and 10 mg/kg body weight nano-TiO_2_ of fresh solutions). The mice were weighed, and the fresh nano-TiO_2_ suspensions within 30 min were administered to the mice by intragastric administration every day for 90 days. Any symptom or mortality was observed and recorded carefully everyday during the 90 days.

After the 90-day period, all mice were weighed and then sacrificed after being anesthetized with ether. Blood samples were collected from the eye vein by rapidly removing the eyeball. Serum was collected by centrifuging blood at 2500 rpm for 10 min. The ovaries of all animals were quickly removed and placed on ice and then dissected and frozen at −80°C except for 40 ovaries for histopathological examination, respectively.

### Mating of Animals

To evaluate the effect of nano-TiO_2_ on the fertility and growth of newborns, we treated three groups of treated female mice (10 in each mating group) for 90 days. After last day of nano-TiO_2_ administration, 10 male and 10 control or treated female mice from each group were put in a common cage for mating. The number of newborns from each pregnant mouse were counted and weighed.

### Relative Weight of Ovary

After weighing the body and ovary, the relative weight of ovary was calculated as the ratio of ovary (wet weight, mg) to body weight (g).

### Titanium Content Analysis

The ovaries were removed from the freezer (−80°C) and thawed. Approximately 0.1 g of the ovary was weighed, digested, and analyzed for titanium content. Inductively coupled plasma-mass spectrometry ([ICP-MS] Thermo Elemental X7; Thermo Electron Co., USA) was used to analyze titanium concentration in the samples.

### Hematological Parameters Determination

Blood samples were collected in tubes containing EDTA as anticoagulant. Red blood cells (RBC), lymphocytes (LYMPH), reticulocytes (Ret), white blood cells (WBC), haemoglobin (HGB) were measured using a hematology autoanalyzer (Cell-DYN 3700).

### Serum Parameters Analysis

Biochemical parameters were evaluated by serum levels of alanine aminotransferase (ALT), aspartate aminotransferase (AST), alkaline phosphatase (ALP), lactate dehydrogenase (LDH), uric acid (UA), blood urea nitrogen (BUN), creatinine (Cr). All biochemical assays were performed using a clinical automatic chemistry analyzer (Type 7170A, Hitachi, Japan).

### Sex Hormone Assays

Sex hormones were evaluated with serum levels of estradiol (E_2_), progesterone (P_4_), luteinizing hormone (LH), follicle stimulating hormone (FSH), prolactin (PRL), testosterone (T), and sex hormone binding globulin (SHBG) using commercial kits (Bühlmann Laboratories, Switzerland). All biochemical assays were performed using a clinical automatic chemistry analyzer (Type 7170A; Hitachi Co., Japan).

### Histopathological Examination of Ovary

For pathologic studies, all histopathologic examinations were performed using standard laboratory procedures. The ovaries were embedded in paraffin blocks, then sliced (5 µm thickness) and placed onto glass slides. After hematoxylin–eosin (HE) staining, the stained sections were evaluated by a histopathologist unaware of the treatments, using an optical microscope (Nikon U-III Multi-point Sensor System, Japan).

### Confocal Raman Microscopy in Ovarian Sections

Raman analysis was performed using backscattering geometry in a confocal configuration at room temperature in a HR-800 Raman microscope system equipped with a 632.817 nm HeNe laser (JY Co., France). Laser power and resolution were approximately 20 mW and 0.3 cm^−1^, respectively, while the integration time was adjusted to 1 s. Ovaries were embedded in paraffin blocks, then sliced into 5 µm in thickness and placed onto glass slides. The slides were dewaxed, hydrated, and then scanned under the confocal Raman microscope.

### Expression Assay of Cytokines

The levels of mRNA expressions of insulin-like growth factor-1 (IGF-1), insulin-like growth factor-binding protein 2 (IGFBP-2), epidermal growth factor (EGF), tumor necrosis factor (TNF-α), tissue plasminogen activator (tPA), luteinizing hormone receptor(LHR), inhibin-α (INH-α), interleukin-1β (IL-1β), IL–6, Fas, Fas ligand (FasL), and growth differentiation factor 9 (GDF-9) in mouse ovary tissue were determined using real-time quantitative RT polymerase chain reaction (RT-PCR) [22]–[24]. Synthesized cDNA was used for the real-time PCR by employing primers that were designed using Primer Express Software according to the software guidelines, and PCR primer sequences are available upon request. To determine levels of protein expressions of IGF- 1, IGFBP-2, EGF, TNF-α, tPA, LHR, INHA, IL-1, IL –6, Fas, FasL, and GDF-9 in the mouse ovary tissue, ELISA was performed using commercial kits that are selective for each respective protein (R&D Systems, USA). Manufacturer’s instruction was followed. The absorbance was measured on a microplate reader at 450 nm (Varioskan Flash, Thermo Electron, Finland), and the concentrations of IGF-1, IGFBP-2, EGF, TNF-α, tPA, LHR, INHA, IL-1β, IL–6, Fas, FasL, and GDF-9 were calculated from a standard curve for each sample.

### Statistical Analysis

All results are expressed as means ± standard error (SE). The significant differences were examined by unpaired Student's t-test using SPSS 19 software (USA). A p-value <0.05 was considered as statistically significant.

## Results

### Body Weight, Relative Weight of Ovary and Titanium Accumulation

The body weight, relative weight of ovary, titanium accumulation in the mouse ovary caused by exposure to nano-TiO_2_ for 90 consecutive days are exhibited in Figs. 1, 2, respectively. It can be seen that with increased nano-TiO_2_ doses, the body weight (Fig. 1 a) and relative weight of ovary (Fig. 1 b) were significantly decreased (P<0.05 or P<0.01), while titanium contents in the ovary were significantly increased (Fig. 2, P<0.01).

**Figure 1:** Changes of body weight and relative weight of ovary of mice caused by intragastric administration of nano-TiO_2_ for 90 consecutive days. Different letters indicate significant differences between groups (p<0.05). Values represent means ± SE (N = 10).

**Figure 2:** Titanium accumulation in mouse ovary caused by intragastric administration of nano-TiO_2_ for 90 consecutive days. Different letters indicate significant differences between groups (p<0.05). Values represent means ± SE (N = 5).

### Hematological and Biochemical Parameters

Results of hematological detection indicate that WBC, LYMPH, NEUT, RBC, and HGB in the nano-TiO_2_-treated female mice were significantly reduced with increased exposure doses (P<<0.05 or p<0.01, Table 1). It can be also seen from Table 1 that nano-TiO_2_ exposure significantly increased the activities of ALT, AST, ALP, LDH, and the levels of Cr, and reduced UA and BUN in sera (P<<0.05 or p<0.01, Table 1), respectively.

**Table 1:** Hematological and biochemical parameters in female mice by intragastric administration of nano-TiO_2_ for 90 consecutive days.

Index	Nano-TiO_2_ (mg/kg BW)			
	0	2.5	5	10
**WBC (10^9^/L)**	7.88±0.39a	5.78±0.29b	4.08±0.20c	2.76±0.14d
**LYMPH** **(10^9^/L)**	6.05±0.30a	3.79±0.19b	2.29±0.11c	1.68±0.08d
**NEUT (10^9^/L)**	1.62±0.08a	1.18±0.06b	0.81±0.04c	0.52±0.03d
**RBC (10^12^/L)**	9.45±0.47a	8.57±0.43b	7.59±0.38c	6.89±0.34d
**HGB (g/L)**	146.12±7.30a	131.55±6.60b	127.11±6.40b	116.55±5.9c
**ALT (U/L)**	19.29±0.96a	22.53±1.13b	26.38±1.32c	35.82±1.79d
**AST (U/L)**	77.27±3.86a	86.25±4.31b	97.56±4.88c	115.39±5.77d
**ALP (U/L)**	92.81±4.64a	108.66±5.43b	118.61±5.93c	136.86±6.84d
**LDH (U/L)**	659.66±32.98a	715.38±35.77b	796.71±39.84c	896.79±44.84d
**UA(µmol/L)**	228.76±11.44a	157.39±7.87b	105.26±5.26c	89.87±0.49d
**Cr (µmol/L)**	8.45±0.422a	9.89±0.49b	12.23±0.61c	14.68±0.73d
***BUN (mmol/L)***	9.56±0.48a	8.02±0.40b	6.88±0.34c	6.05±0.30d

Different letters indicate significant differences between groups (p<0.05). Values represent means ± SE (N = 5).

### Reproduction

With increased nano-TiO_2_ exposed doses, decreased mating rate, pregnancy rate, number of newborns and weight of neonates of mice were significantly observed in Table 2 (P<0.05). In addition, nano-TiO_2_ led to reduction of survival of young mice at 28th day after birth (P<0.05).

**Table 2:** Effects of nano-TiO_2_ on conception of female mice, number of newborns, and weight of neonates after intragastric administration of nano-TiO_2_ for 90 consecutive days.

Index	Nano-TiO_2_ (mg/kg BW)			
	0	2.5	5	10
**Mating rate (%)**	100±5a	85±4.25b	75±3.75c	65±3.25d
**Pregnancy rate (%)**	100±5a	81±4.05b	72±3.6c	58±2.90d
**Number of newborns**	14±0.7a	10±0.5b	8±0.4c	6±0.3d
**Weight of neonates female mice in 1st** **after birth (g)**	1.54±0.077a	1.52±0.076a	1.45±0.073b	1.40±0.07b
**Weight of neonates male mice in 1st** **after birth (g)**	1.57±0.079a	1.54±0.077a	1.47±0.074b	1.41±0.07b
***Survival rate of young mice in 28th day*** ***after birth (%)***	98±4.90a	89±4.45b	81±4.05c	72±3.60d

Different letters indicate significant differences between groups (p<0.05). Values represent means ± SE (N = 5).

### Sex Hormone Levels

As shown in Table 3, serum E2 levels were gradually increased (P<0.05), contrary, P4, LH, FSH, and T were significantly decreased in female mice (P<0.05) with increased nano-TiO_2_ exposed doses. However, no significant differences between serum PRL and SHBG levels in the nano-TiO_2_ exposed female mice and those of control were observed (P>0.05).

**Table 3:** Effects of nano-TiO_2_ on sex hormone levels in sera of female mice.

Hormone level	Nano-TiO_2_ NPs (mg/kg BW)			
	0	2.5	5	10
**E2 (pmol/L)**	83.66±4.18a	91.09±4.554b	101.98±5.10c	111.88±5.59d
**P4 (nmol/L)**	34.99±1.75a	30.11±1.506b	26.49±1.32c	23.42±1.17d
**LH (IU/L)**	0.12±0.006a	0.061±0.003b	0.038±0.002c	0.021±0.001d
**FSH (IU/L)**	0.48±0.024a	0.42±0.021b	0.37±0.018c	0.28±0.014d
**PRL (µg/L)**	0.60±0.030a	0.64±0.032a	0.67±0.033a	0.73±0.036a
**T (ng/dL)**	71.13±3.56a	61.55±3.08b	55.01±2.75c	49.02±2.45d
***SHBG (nmol/L)***	0.43±0.021a	0.42±0.021a	0.42±0.021a	0.42±0.021a

Different letters indicate significant differences between groups (p<0.05). Values represent means ± SE (N = 5).

### Histopathological Evaluation

Figure 3 presents histological changes in ovary. Normal development of primary follicle and secondary follicle from the control ovary was observed (Fig. 3 a, b). In the nano-TiO_2_-treated groups, however, a large of atretic follicles, severe inflammatory cell infiltration, and necrosis were observed (Fig. 3 d–e), respectively. In addition, we also observed significant black agglomerates in the ovary samples exposed to 10 mg/kg of nano-TiO_2_ (Fig. 3e). Confocal Raman microscopy further showed a characteristic nano-TiO_2_ peak in the black agglomerate (148 cm^−1^), which further confirmed the deposition of nano-TiO_2_ in the ovary (see spectrum B in the Raman insets in Fig. 3f). The results also suggest that exposure to nano-TiO_2_ dose-dependently deposited in the ovary, thus severely resulted in the ovarian injuries.

**Figure 3:** Histopathological observation of ovary of mice caused by intragastric administration of nano-TiO_2_ for 90 consecutive days. (a) control groups (unexposed mice) present normal development of primary follicle and secondary follicle; (b) 2.5 mg/kg nano-TiO_2_-exposed group: green cycle suggest inflammatory cell infiltration, yellow arrows indicate atretic follicle, red arrows present apoptosis or tissue necrosis; (c) 5 mg/kg nano-TiO_2_-exposed group: green cycle suggest severe inflammatory cell infiltration, yellow cycles present nano-TiO_2_ deposition, yellow arrows indicate atretic follicle, red arrows present apoptosis or tissue necrosis in ovary; (d) 10 mg/kg nano-TiO_2_ -exposed group: green cycle suggest severe inflammatory cell infiltration, yellow arrows indicate atretic follicle, red arrows present tissue necrosis, yellow cycle may show aggregation of nano-TiO_2_ in ovary. Arrow A spot is a representative cell that not engulfed the nano-TiO_2_, while arrow B spot denotes a representative cell that loaded with nano-TiO_2_. The right panels show the corresponding Raman spectra identifying the specific peaks at about 148 cm^−1^.

### Cytokines Expression

To confirm molecular mechanisms of nano-TiO_2_ on the ovary injury, the expression of the inflammation-related genes or follicular atresia-related genes and their proteins in the ovary were examined (Tables 4, 5). It can be observed that exposure to nano-TiO_2_ resulted in significant increases of IGFBP-2, EGF, TNF-α, tPA, IL-1β, IL –6, Fas, and FasL expression, while obviously decreased IGF-1, LHR, INH-α, and GDF-9 expression in the ovary compared with the control (P<0.05 or 0.01), which are consistent with the trends of fertility reduction and ovary injury.

**Table 4:** Effect of nano-TiO_2_ on the levels of cytokine gene mRNA expression in mouse ovary.

Ratio ofgene/actin	Nano-TiO_2_ (mg/kg BW)			
	0	2.5	5	10
***IGF-1/actin***	1.35±0.068a	0.92±0.046b	0.58±0.029c	0.32±0.016d
***IGFBP-2/actin***	0.41±0.021a	0.69±0.035b	0.99±0.050c	1.37±0.069d
***EGF/actin***	0.71±0.036a	1.03±0.052b	1.38±0.069c	1.75±0.088d
***TNF-α/actin***	0.27±0.014a	0.43±0.022b	0.69±0.035c	0.97±0.049d
***tPA/actin***	0.07±0.004a	0.28±0.014b	0.42±0.021c	0.56±0.028d
***LHR/actin***	0.46±0.023a	0.25±0.013b	0.12±0.006c	0.05±0.003d
***INH-α/actin***	0.95±0.048a	0.61±0.031b	0.38±0.019c	0.12±0.006d
***IL-1β/actin***	0.22±0.011a	0.39±0.020b	0.68±0.034c	1.05±0.053d
***IL-6/actin***	0.09±0.005a	0.25±0.013b	0.48±0.024c	0.76±0.038d
***Fas/actin***	0.55±0.028a	0.78±0.039b	1.06±0.053c	1.67±0.084d
***FasL/actin***	0.33±0.017a	0.54±0.027b	0.86±0.043c	1.13±0.057d
***GDF-9/actin***	1.07±0.054a	0.72±0.036b	0.46±0.023c	0.29±0.015d

Different letters indicate significant differences between groups (p<0.05). Values represent means ± SE (N = 5).

**Table 5:** Effects of nano-TiO_2_ on the levels of cytokine protein expression in mouse ovary.

Protein expression (ng/g tissue)	Nano-TiO_2_ (mg/kg BW)			
	0	2.5	5	10
**IGF-1**	117.62±5.88a	92.29±4.61b	74.19±3.71c	61.24±3.06d
**IGFBP-2**	34.38±1.72a	40.41±2.02b	47.30±2.36c	61.61±3.08d
**EGF**	41.22±2.06a	65.38±3.27b	82.85±4.14c	102.42±5.12d
**TNF-α**	20.00±1.00a	31.03±1.75b	50.14±2.51c	71.49±3.57d
**tPA**	11.32±0.56a	18.50±0.93b	26.44±1.32c	34.22±1.71d
**LHR**	39.53±1.98a	29.73±1.49b	21.76±1.09c	15.21±0.76d
**INH-α**	82.90±4.14a	66.77±3.34b	52.18±2.61c	38.85±1.94d
**IL-1β**	22.98±1.15a	30.52±1.53b	38.20±1.91c	47.38±2.37d
**IL-6**	10.99±0.55a	19.19±0.96b	31.59±1.58c	42.04±2.10d
**Fas**	43.37±2.17a	64.47±3.22b	89.99±4.50c	125.98±6.30d
**FasL**	31.45±1.57a	42.24±2.11b	54.05±2.70c	67.11±3.35d
***GDF-9***	85.37±4.27a	66.70±3.33b	47.85±2.39c	31.19±1.56d

Different letters indicate significant differences between groups (p<0.05). Values represent means ± SE (N = 5).

## Discussion

To confirm effects of reproductive system of female mice caused by 90 consecutive days exposure to low dose of nano-TiO_2_, the present study was designed to investigate the changes of ovarian morphology, fertility, hormone levels and expression of relevant genes and their proteins in mouse ovary.

Our findings indicated that the oral nano-TiO_2_ with 2.5, 5, and 10 mg/kg BW doses for 90 consecutive days led to atretic follicle increases, severe inflammatory response and necrosis in the ovary (Fig. 3). Increased atretic follicles were closely associated with premature ovarian failure following nano-TiO_2_–induced toxicity. Furthermore, the present study also suggested that exposure to nano-TiO_2_ reduced mating rate, pregnancy rate, number of newborns and growth of neonates (Table 2) and altered sex hormone levels, including a significant increase of E2 concentration and great decreases of P4, LH, FSH, and T concentrations in the sera (Table 3). Decreased mating capacity of female mice following exposure to nano-TiO_2_ may be associated with imbalance of sex hormone levels. Follicular atresia is not only the break-down of the ovarian follicles, but also is hormonally controlled apoptosis.Therefore, FSH and LH reduction by exposure to nano-TiO_2_ resulted in the follicular atresia in mouse ovary. Theoretically, increased effect on E2 levels may be due to the activation of cytochrome P450 aromatase, which converts T into E2 [25]. Elevated E2 and decreased T caused by nano-TiO_2_ may be related to activate cytochrome P450 aromatase, promoting transformation from T to E2, but it needs to study in future. Taken together, increased atretic follicles and decreased fertility were due to reduction of FSH, P_4_, LH, and T levels in the nano-TiO_2_ treated female mice. In addition, T has wide ranging roles in ovarian function, including granulosa cells, theca cells, oocytes, and interstitial cells, because T enhances IGF-I and IGF-I receptor mRNAs in primates [26]. Activins, inhibins, GDF-9, and TGF-β of growth and differentiation factors can influence follicular development [27]. Therefore, the ovarian injuries and changes of sex hormone levels in female mice may be due to nano-TiO_2_ alter the expression of relevent genes and their proteins in the ovary. To identify the mechanisms of multiple cytokines working together caused by nano-TiO_2_, mRNA and protein expression of IGFBP-2, EGF, TNF-α, tPA, LHR, INH-α, IL-1β, IL–6, Fas, FasL and GDF-9 from ovary were examined. The assays indicated that the levels of these cytokines were significantly altered (Tables 4, 5). The main results are discussed below.

In mammals, most of ovarian follicles undergo atresia during development, and only a few differentiate to mature finally. Apoptosis occurs in ovarian follicular granulosa cell of majority of animals during follicular atesia, which is the cause of atretic initiation and progression [28]. Therefore apoptosis is suggested to regulated by various factors and atretogenic factors [29]. Intrafollicular IGF-1 plays a critical role in the enhanced response (estradiol production) of the future dominant follicle to the small rise in FSH that initiates the follicular wave. The binding of IGF to its receptors is strongly modulated by a family of six high-affinity IGF-binding proteins (IGFBPs). IGFBP-2 inhibits IGF effect on gonadotropin-induced follicular growth and differentiation. EGF is involved in regulation of ovarian cell proliferation and differentiation. So, EGF, IGF-1 and gonadotropins are determined to be survival factors, but IGFBPs are atretogenic factors [30]. Luo and Zhu demonstrated that FSH concentration, and IGF-1 expression were decreased, contrary IGFBP-2 and EGF expression were increased in process of induced follicular atresia of female rat [31]. Our data indicated that the levels of IGFBP-2 and EGF expression were significantly elevated, whereas IGF-1 expression was greatly inhibited in the nano-TiO_2_–treated ovary (Tables 4, 5), suggesting that follicular atresia caused by nano-TiO_2_ (Fig. 3) may be involved in increased IGFBP-2 and EGF, and decreased IGF-1 in the ovary.

Granulosa cells produce estrogen which can synergistically promote FSH-induced self-production of LHR and aromatase activity in cells. In contrast to estrogen, androgen is capable of inducing follicular atresia. Inhibin has also been demonstrated to be an atretic factor. To form bioactive dimers linked by disulfate bonds, one α subunit combines with one of the two β subunits will form two types of inhibin, and combination of two types of β subunits will form three types of actin. Inhibin and actin are involved in coordination between gonadotropins or other factors in regulation of follicular selection, development and atesia [32]. tPA is responsible for the cumulus cell expansion, dispersion and oocyte maturation. Yan et al indicated that tPA expression was significantly increased, but LHR and inhibin subunits were not expressed in the follicle undergoing atresia in rats [33]. Our findings also showed that nano-TiO_2_ greatly promoted tPA expression, but inhibited LHR and INH-α expression in the ovary (Tables 4, 5), which may lead to follicular atresia in female mice (Fig. 3).

It had been suggested that Fas can be not only found in murine oocytes obtained from atretic follicles [34], but also in granulosa cells of follicles undergoing atresia in the ovary [35]. FasL was also demonstrated to express in the granulosa cells and antral atretic follicles from rat [35], and in granulosa cells of atretic follicles from mouse ovary [36]. Fas and FasL expression in the ovary raise the possibility of Fas-FasL interaction as a mediator of apoptosis during follicular atresia [37]. In the present study, the significant increases of Fas and FasL expression in the ovary are observed following nano-TiO_2_ induced toxicity (Tables 4, 5), which may conduct to atretic follicle formation of female mice (Fig. 3).

As we know, TNF-α induces apoptosis in several cellular models, and is produced locally in the rat, ovine ovarian granulosa cells and oocytes, and may act as a paracrine regulatory factor [38]. IL- 1β, IL-6 and androgens produced locally in the ovary are also demonstrated to induce follicular atresia [39]. GDF-9 is a growth factor secreted by oocytes in growing ovarian follicles, which is essential for normal follicular development [27]. GDF-9-deficient female mice are infertile because of an early block in folliculogenesis at the type 3b primary follicle stage [40]. Increased levels of TNF-α, IL-1β and IL–6 expressions are also demonstrated to be closely associated with inflammation generation in human and animals. The previous studies suggested that expressions of TNF-α, IL-1β and IL–6 were significantly elevated in the nano-TiO_2_ exposed lung [41]–[44], liver [45]–[49], kidney [5], [8], [50], and spleen [5], [19], [51]–[53] of animals. The present findings showed that nano-TiO_2_ exposure markedly promoted expression of TNF-α, IL-1β and IL –6, but significantly inhibited GDF-9 expression in mouse ovary (Tables 4, 5), which resulted in inflammation and follicular atresia in mouse ovary (Fig. 3). A scheme that links the nano-TiO_2_ and the changes of IGFBP-2, IGF-1, EGF, tPA, LHR, INH-α, Fas, FasL, GDF-9, TNF-α, IL-1β, and IL –6 is depicted in Figure 4.

**Figure 4:** A schematic showing possible mechanisms of nano-TiO_2_ induced follicular atresia in mouse ovary.

## Conclusion

In the present study, we demonstrate that the exposure to nano-TiO_2_ could result in the fertility reduction, ovarian inflammation and follicaular atresia in a dose-dependent manner, which were closely related to reduction of immunity, biochemical dysfunction, imbalance of sex hormones, and changes of IGFBP-2, IGF-1, EGF, tPA, LHR, INH-α, Fas, FasL TNF-α, IL-1β, IL –6, and GDF-9 expressions in the ovary. Therefore, our findings suggested the need for great caution to handle the nanomaterials for workers and consumers.

## References

[1] Fisher J, Egerton T (2001) Titanium Compounds, Inorganic. Kirk-Othmer Encyclopedia of Chemical Technology. John Wiley & Sons, New York.

[2] KaidaT, KobayashiK, AdachiM, SuzukiF (2004) Optical characteristics of titanium oxide interference film and the film laminated with oxides and their applications for cosmetics. J Cosmet Sci 55: 219–220.15190897

[3] Esterkin CR, Negro AC, Alfano OM, Cassano AE (2005) Air pollution remediation in a fixed bed photocatalytic reactor coated with TiO_2_. AIChE J 51, 2298–2310.

[4] ChoiH, StathatosE, DionysiouDD (2006) Sol–gel preparation of mesoporous photocatalytic TiO_2_ films and TiO_2_/Al_2_O_3_ composite membranes for environmental applications. Appl Catal B – Environ 63: 60–67.

[5] ChenJY, DongX, ZhaoJ, TangGP (2009) In vivo acute toxicity of titanium dioxide nanoparticles to mice after intraperitoneal injection. J Appl Toxicol 29: 330–337.1915671010.1002/jat.1414

[6] ScownTM, van AerleRY, JohnstonBD, CumberlandS, LeadJR, et al (2009) High doses of intravenously administered titanium dioxide nanoparticles accumulate in the kidneys of rainbow trout but with no observable impairment of renal function. Toxicol Sci 109: 372–380.1933265010.1093/toxsci/kfp064

[7] ZhaoJF, WangJ, WangSS, ZhaoXY, YanJY, et al (2010) The mechanism of oxidative damage in nephrotoxicity of mice caused by nano-anatase TiO_2_ . J Exp Nanosci 5: 447–462.

[8] GuiSX, ZhangZL, ZhengL, CuiYL, LiuXR, et al (2011) Molecular mechanism of kidney injury of mice caused by exposure to titanium dioxide nanoparticles. J Hazard Mater 195: 365–370.2190748910.1016/j.jhazmat.2011.08.055

[9] Yu Y, Ren W, Ren B (2008) Nanosize titanium dioxide cause neuronal apoptosis: A potential linkage between nanoparticle exposure and neural disorder. Neurol Res doi: 10.1179/17431 3208X 305391.10.1179/0161641215Z.00000000058726154883

[10] WuJ, LiuW, XueCB, ZhouSC, LanFL, et al (2009) Toxicity and penetration of TiO_2_ nanoparticles in hairless mice and porcine skin after subchronic dermal exposure. Toxicol Lett 2191: 1–8.10.1016/j.toxlet.2009.05.02019501137

[11] MaLL, LiuJ, LiN, WangJ, DuanYM, et al (2010) Oxidative stress in the brain of mice caused by translocated nanoparticulate TiO_2_ delivered to the abdominal cavity. Biomaterials 31: 99–105.1978329610.1016/j.biomaterials.2009.09.028

[12] HuRP, GongXL, DuanYM, LiN, CheY, et al (2010) Neurotoxicological effects and the impairment of spatial recognition memory in mice caused by exposure to TiO_2_ nanoparticles. Biomaterials 31: 8043–8050.2069269710.1016/j.biomaterials.2010.07.011

[13] HuRP, ZhengL, ZhangT, CuiYL, GaoGD, et al (2011) Molecular mechanism of hippocampal apoptosis of mice following exposure to titanium dioxide nanoparticles. J Hazard Mater 191: 32–40.2157017710.1016/j.jhazmat.2011.04.027

[14] ShinJA, LeeEJ, SeoSM, KimHS, KangJL, et al (2010) Nanosized titanium dioxide enhanced inflammatory responses in the septic brain of mouse. Neurosci 165: 445–454.10.1016/j.neuroscience.2009.10.05719892005

[15] GuoLL, LiuXH, QinDX, GaoLL, ZhangHM, et al (2009) Effects of nanosized titanium dioxide on the reproductive system of male mice. National J Androl15(6): 517–522 (abstract in English)..19593991

[16] HouJ, WanXY, WangF, XuGF, LiuZ, et al (2009) Effects of titanium dioxide nanoparticles on development and maturation of rat preantral follicle in vitro. Academ J Second Milit Med Univ 30(8): 869–873 (abstract in English)..

[17] LiuR, YuanQL, FanCJ, YinLH, PuYP (2009) Toxicity of TiO_2_ nanoparticles on nematode Caenorhabditis elegans. Ch in J Public Health 25(3): 310–312 (abstract in English)..

[18] Di VirgilioAL, ReigosaM, ArnalPM, Fernández Lorenzo de MeleM (2010) Comparative study of the cytotoxic and genotoxic effects of titanium oxide and aluminium oxide nanoparticles in Chinese hamster ovary (CHO-K1) cells. J Hazard Mater 177: 711–718.2007996810.1016/j.jhazmat.2009.12.089

[19] WangJ, LiN, ZhengL, WangY, DuanYM, et al (2011) P38-Nrf-2 signaling pathway of oxidative stress in mice caused by nanoparticulate TiO_2_ . Biol Trace Elem Res 140: 186–197.2042231110.1007/s12011-010-8687-0

[20] TakedaK, SuzukiK, IshiharaA, Kubo-IrieM, FujimotoR, et al (2009) Nanoparticles transferred from pregnant mice to their offspring can damage the genital and cranial nerve systems. J Health Sci 55(1): 95–102.

[21] YangP, LuC, HuaN, DuY (2002) Titanium dioxide nanoparticles co-doped with Fe^3+^ and Eu^3+^ ions for photocatalysis. Mater Lett 57: 794–801.

[22] KeLD, ChenZ (2000) A reliability test of standard-based quantitative PCR: exogenous vs endogenous standards. Mol. Cell Probes 14: 127–135.10.1006/mcpr.2000.028810799275

[23] LivakKJ, SchmittgenTD (2001) Analysis of relative gene expression data using real-time quantitative PCR and the 2(-Delta Delta C(T)) method. Methods 25: 402–408.1184660910.1006/meth.2001.1262

[24] LiuWH, SaintDA (2002) Validation of a quantitative method for real time PCR kinetics. Biochem. Biophys Res Commun 294: 347–353.10.1016/S0006-291X(02)00478-312051718

[25] AugerAP, TetelMJ, McCarthyMM (2000) Steroid receptor coactivator-1 (SRC-1) mediates the development of sex-specific brain morphology and behavior. Proc Natl Acad Sci USA 97: 7551–7555.1086101810.1073/pnas.97.13.7551PMC16583

[26] VendolaKA, ZhouJ, WangJ, FamuyiwaOA, BievreM, et al (1999) Androgens promote oocyte insulin-like growth factor 1 expression and initiation of follicle development in the primate ovary. Biol Reprod 61: 353–357.1041151110.1095/biolreprod61.2.353

[27] DongJ, AlbertiniDF, NishimoriK, KumarTR, LuN, et al (1996) Growth differentiation factor-9 is required during early ovarian folliculogenesis. Nature 383: 531–535.884972510.1038/383531a0

[28] ManikkamM, RajamahendranR (1997) Progesterone-induced atresia of the proestrous dominant follicle in the bovine ovary: Changes in diameter, insulin-like growth factor system, aromatase activity, steroid hormones, and apoptotic index. Biol Reprod 57: 580–587.928299410.1095/biolreprod57.3.580

[29] HsuehAJW, BilligH, TsafririA (1994) Ovarian Follicle Atresia: A Hormonally Controlled Apoptotic Process. Endocr Rev 15(6): 707–724.770527810.1210/edrv-15-6-707

[30] ChunSY, BilligH, TillyJL, FurutaI, TsafririA, et al (1994) Gonadotropin suppression of apoptosis in cultured preovulatory follicles: mediatory role of endogenous insulin-like growth factor I. Endocrinol. 135(5): 1845–1853.10.1210/endo.135.5.75252557525255

[31] LuoWX, ZhuC (2000) Expression and regulation of mRNAs for insulin-like growth factor (IGF-1), IGF-binding protein-2, and LH receptor in the process of follicaular atresia. Sci in Chi, Ser C 43(3): 272–279.10.1007/BF0287928618726382

[32] FindlayJK (1993) An update on the roles of inhibin, activin, and follistatin as local regulators of folliculogenesis. Biol Reprod 48: 15–23.841890310.1095/biolreprod48.1.15

[33] YanJL, FengQ, LiuHZ, FuGQ, LiuYX (1999) Expression of tPA, LH recptor and inhibin α, β_A_ subunits during follicular atresia in rat. Sci in Chin, Ser C 42(6): 583–590.10.1007/BF0288157518726480

[34] GuoMW, MoriE, XuJP, MoriT (1994) Identification of Fas antigen associated with apoptotic cell death in murine ovary. Biochem Biophys Res Commun 203: 1438–1446.752448410.1006/bbrc.1994.2346

[35] KimJM, YoonYD, TsangBK (1999) Involvement of the Fas/Fas ligand system in p53-mediated granulosa cell apoptosis during follicular development and atresia. Endocrinol 140: 2307–2317.10.1210/endo.140.5.672610218984

[36] GuoMW, XuJP, MoriE, SatoE, SaitoS, et al (1997) Expression of Fas ligand in murine ovary. Am J Reprod Immunol 37: 391–398.919679810.1111/j.1600-0897.1997.tb00249.x

[37] Andreu-VieyraCV, HabibiHR (2000) Factors controlling ovarian apoptosis. Can J Physiol Pharmacol 78: 1003–1012.11149378

[38] MurdochWJ, ColginDC, EllisJA (1997) Role of tumor necrosis factor alpha in the ovulatory mechanism of ewes. J Anim Sci 75: 1601–1605.925052310.2527/1997.7561601x

[39] KaipiaA, HsuehAJW (1997) Regulation of ovarian follicle atresia. Annu Rev Physiol 59: 349–363.907476810.1146/annurev.physiol.59.1.349

[40] ElvinJA, YanC, WangP, NishimoriK, MatzukMM (1999) Molecular characterization of the follicle defects in the growth differentiation factor-9-deficient ovary. Mol Endocrinol 13(6): 1018–1034.1037989910.1210/mend.13.6.0309

[41] ChenHW, SuSF, ChienCT, LinWH, YuSL, et al (2006) Titanium dioxide nanoparticles induce emphysema-like lung injury in mice. FASEB J 20: 1732–1741.10.1096/fj.06-6485fje17023518

[42] HougaardKS, JacksonP, JensenKA, SlothJJ, LoschnerK, et al (2010) Effects of prenatal exposure to surface-coated nanosized titanium dioxide (UV-Titan). A study in mice. Part Fibre Toxicol 7: 16.2054655810.1186/1743-8977-7-16PMC2908059

[43] SunQQ, TanDL, ZhouQP, LiuXR, ChengZ, et al (2012) Oxidative damage of lung and its protective mechanism in mice caused by long-term exposure to titanium dioxide nanoparticles. J Biomed Mater Res A 100(10): 2554–2562.2252876010.1002/jbm.a.34190

[44] SunQQ, TanDL, ZeYG, SangXZ, LiuXR, et al (2012) Pulmotoxicological effects caused by long-term titanium dioxide nanoparticles exposure in mice. J Hazard Mater 235–236: 47–53.10.1016/j.jhazmat.2012.05.07222898172

[45] MaLL, ZhaoJF, WangJ, DuanYM, LiuJ, et al (2009) The acute liver injury in mice caused by nano-anatase TiO_2._ . Nanosacle Res Lett 4: 1275–128.10.1007/s11671-009-9393-8PMC289409020628458

[46] CuiYL, GongXL, DuanYM, LiN, HuRP, et al (2010) Hepatocyte apoptosis and its molecular mechanisms in mice caused by titanium dioxide nanoparticles. J Hazard Mater 183: 874–880.2072406710.1016/j.jhazmat.2010.07.109

[47] CuiYL, LiuHT, ZhouM, DuanYM, LiN, et al (2011) Signaling pathway of inflammatory responses in the mouse liver caused by TiO_2_ nanoparticules. J Biomed Mater Res A 96(1): 221–229.2110517110.1002/jbm.a.32976

[48] CuiYL, HuitingLiu, ZeYG, ZhangZL, HuYY, et al (2012) Gene expression in liver injury caused by long-term exposure to titanium dioxide nanoparticles in mice. Toxicol Sci 128(1): 171–185.2253962310.1093/toxsci/kfs153

[49] JacksonP, HalappanavarS, HougaardKS, WilliamsA, MadsenAM, et al (2013) Maternal inhalation of surface-coated nanosized titanium dioxide (UV-Titan) in C57BL/6 mice: effects in prenatally exposed offspring on hepatic DNA damage and gene expression. Nanotoxicol 7: 85–96.10.3109/17435390.2011.63371522117692

[50] WangJX, ZhouGQ, ChenCY, YuHW, WangTC, et al (2007) Acute toxicity and biodistribution of different sized titanium dioxide particles in mice after oral administration. Toxicol Lett 168: 176–185.1719713610.1016/j.toxlet.2006.12.001

[51] LiN, DuanYM, HongMM, ZhengL, FeiM, et al (2010) Spleen injury and apoptotic pathway in mice caused by titanium dioxide nanoparticules. Toxicol Lett 195: 161–168.2038159510.1016/j.toxlet.2010.03.1116

[52] WangJX, ZhuXS, ZhangXZ, ZhaoZ, LiuHA (2011) Disruption of zebrafish (Danio rerio) reproduction upon chronic exposure to TiO_2_ nanoparticles. Chemosphere 83: 461–467.2123903810.1016/j.chemosphere.2010.12.069

[53] SangXZ, ZhengL, SunQQ, ZhangT, LiN, et al (2012) The chronic spleen injury of mice following exposure to titanium dioxide nanoparticules. J Biomed Mater Res Part A 100(4): 894–902.10.1002/jbm.a.3402422275130

